# Analysis of the Effect of Cluster Nursing in Postoperative Hypertensive Cerebral Hemorrhage

**DOI:** 10.1155/2021/3448979

**Published:** 2021-12-02

**Authors:** Pingxia Zheng, Jia Wang, Yan Ma, Jingjing Xu, Qianping Zhu

**Affiliations:** ^1^Department of Thoracic Surgery, Zhejiang Hospital, Hangzhou 310012, Zhejiang, China; ^2^Brain Center, Zhejiang Hospital, Hangzhou 310012, Zhejiang, China

## Abstract

Hypertensive intracerebral hemorrhage is a common condition in clinic. Due to the improvement of minimally invasive technology, its therapeutic effect is good, but there are still postoperative complications. The corresponding routine nursing intervention is not effective in the rehabilitation of postoperative patients with hypertensive intracerebral hemorrhage. In this paper, cluster nursing was applied to the treatment of postoperative patients with hypertensive intracerebral hemorrhage. For this purpose, a retrospective study or experiment was conducted on 150 patients with hypertensive intracerebral hemorrhage in the hospital specifically from January 2019 to December 2020. According to the nursing strategy, patients were divided into experimental (*n* = 75) and control groups (*n* = 75), respectively. The control group adopted routine nursing mode, whereas the experimental group adopted cluster nursing mode. The treatment compliance of patients in the experimental group was 86.67%, while that in the control group was 73.33% (*P* < 0.05). The total incidence of postoperative complications in the experimental group was 3.2%, which was lower than 25% in the control group (*P* < 0.05). The motor function score of the experimental group was better than that of the control group (*P* < 0.05). The application of cluster nursing in postoperative patients with hypertensive intracerebral hemorrhage is feasible, and its nursing effect is significant, which can not only reduce the incidence of postoperative complications but also improve patients' compliance and quality of life. It has good application value.

## 1. Introduction

Hypertensive intracerebral hemorrhage is a common and frequently occurring condition in clinic. The incidence of hypertensive intracerebral hemorrhage in China accounts for 21%–48% of the total incidence of stroke, and mortality rate ranks first among cerebrovascular diseases [1]. The disease is mainly caused by long-term hypertension leading to vitreous or cellulosic degeneration of the vascular wall of the perforating arterioles in the brain, resulting in intracranial vascular rupture caused by reduced elasticity and strength [2]. With the continuous improvement of medical technology, the mortality of hypertensive intracerebral hemorrhage has been reduced, but the incidence of complications in patients with the disease is still relatively high, seriously affecting the quality of life of patients. It is considered to be one of the most difficult public health problems facing all mankind.

In clinic, the traditional treatment of hypertensive intracerebral hemorrhage is to use large bone flap craniotomy to treat patients with hypertensive intracerebral hemorrhage, which removes hematoma under microscope. The clearance rate of hematoma is higher, so it has great trauma and great damage to normal brain tissue [3]. In recent years, with the development and improvement of minimally invasive technology, ultra-early minimally invasive surgery with small bone window has been widely used in the clinical treatment of patients with hypertensive intracerebral hemorrhage, and its therapeutic effect is good, but there are still postoperative complications [4].

The incidence of postoperative complications of hypertensive intracerebral hemorrhage shows an increasing trend, for example, DVT emboli fall off with the blood circulation to the lungs, which will lead to pulmonary embolism and death, and intestinal dysfunction and bedsores will also lead to the decline of motor function of patients. This limitation of treatment may lead to a decline in patients' confidence in treatment, irritation, and other negative emotions, thus reducing patients' compliance. It has a negative effect on the overall treatment [5, 6]. In the literature, the nursing intervention measures for the prevention of postoperative complications of cerebral hemorrhage are summarized as early monitoring, physical prevention, drug prevention, strengthening management, psychological nursing, and so on, but there is a lack of overall evaluation of patients and no systematic nursing thinking. Nutrition assessment and limb functional exercise and other details are not considered enough [7]. Cluster nursing is a nursing program formed by a series of interrelated interventions with evidence-based basis, which usually includes 3 to 5 simple, clear, and operational evidence-based practical measures. The simultaneous implementation of these measures can better improve the outcome of patients than alone [8].

To resolve the aforementioned issues associated with existing state-of-the-art techniques, a cluster-oriented nursing model is used to nurse the postoperative patients with hypertensive intracerebral hemorrhage and its clinical application value was evaluated. Main contributions of this paper to the scientific community or healthcare research domain are provided in the following.

  A cluster-oriented nursing model was designed and developed to nurse the postoperative patients with hypertensive intracerebral hemorrhage in the traditional hospital.
  A clinical application value was thoroughly evaluated using experimental observations performed in the hospital.
  A retrospective study or experiment was successfully conducted to evaluate its effects on the health status of various patients.
  A uniform classification and selection strategy for patients to be divided into two groups, i.e., control and experimental, was proposed.

The remaining portions of this paper are organized according to the following agenda items which are given as follows.

In subsequent section, the proposed methods along with datasets are defined in such a way that sufficient detail is provided. In Section 3, experimental results and observations are presented in detail, whereas generalized discussion about the proposed scheme and exiting models is provided in the subsequent section. Finally, concluding remarks and future directives are provided.

## 2. Proposed Method

### 2.1. Study Subjects

From January 2019 to December 2019, 75 patients with hypertensive intracerebral hemorrhage were included in the control group, and from January 2020 to December 2020, 75 patients with hypertensive intracerebral hemorrhage were included in the experimental group. These patients were treated surgically, excluding patients with serious diseases such as heart, lung, and kidney, history of cerebral infarction, poor coagulation function, and so on. The average age was (68.45 ± 14.4) years, including 36 female patients and 114 male patients. 75 patients took routine nursing measures, and 75 patients took cluster nursing measures. The nursing results of the two groups were compared to draw a conclusion. There was no significant difference in gender, age, bleeding volume, and bleeding site between the two groups (*P* > 0.05).

### 2.2. Study Methods

The control group was treated with routine nursing, including condition monitoring, medicine, diet, rest guidance, psychological counseling, and health education. The experimental group adopted the cluster nursing model, systematic intervention was carried out in the nursing process, and various links involved in postoperative nursing of patients with hypertensive intracerebral hemorrhage were optimized, and the senior responsible nurses in charge of the bed worked out the cluster nursing plan and trained the nurses in each class; it required the nurses in each class to skillfully master the technical nursing measures. In the process of nursing, it is carried out in strict accordance with the established plan. The program mainly includes basic nursing, specialist nursing, respiratory tract intervention, posture intervention, nutrition intervention, psychological nursing, and quality control. To put it simply, they have to remove the secretions in the patient's mouth in time and take sputum suction measures according to the actual situation of the patient to reduce the stimulation to the respiratory tract; guide the patient to take the lateral position, raise the head of the bed slightly, and help the patient turn over at an interval of 2 hours; keep the skin clean and dry, especially the skin that has been oppressed for a long time, and avoid the occurrence of pressure sores; evaluate the nutritional status of patients, give targeted nutritional support according to the evaluation results, and improve the immune ability of patients; evaluate the psychological needs of patients and then take targeted psychological care to communicate with patients; and establish a good relationship with patients to make patients trust nurses. Responsible nurses analyze whether the plan of cluster nursing is standardized or not and whether patients and family members have mastered the contents of education. The head nurse analyzed whether the implementation of cluster nursing was correct, the result of nursing intervention was ideal, and the effect of improving patients' motor dysfunction was analyzed.

### 2.3. Observation Indicators

#### 2.3.1. Compliance of Patients with Treatment

The treatment compliance of patients with low salt and low-fat diet, taking medicine on time, reasonable exercise, and regular examination was evaluated, which were divided into good compliance and moderate compliance, adhering to long-term standardized treatment in accordance with the doctor's advice. In most cases, the patients could be treated according to the doctor's advice. Patients with poor compliance cannot adhere to long-term treatment or interrupt treatment. Such patients often cannot follow the advice of doctors.

#### 2.3.2. Incidence of Complications

The incidence of postoperative complications including bedsore, pulmonary infection, intestinal dysfunction, and deep venous thrombosis (DVT) was observed and compared between the two groups.

#### 2.3.3. Motor Function Score

According to the Fugl-Meyer motor function rating scale, the motor function of the two groups before and after nursing was evaluated and compared. There were five items in the scale, namely, upper limb, lower limb, limb sensory recovery, balance, and joint activity. The full score was 100, and the score was negatively correlated with the degree of motor dysfunction. <50 points indicated that the patients had severe motor dysfunction, 50∼84 points indicated that the patients had obvious motor dysfunction, 85–95 points indicated that the patients had moderate motor dysfunction, and >96 points indicated that the patients had mild motor dysfunction.

#### 2.3.4. Statistical Methods

SPSS18.0 was used for data statistics, in which *χ*^2^ (%) was used for counting data, and *t*-test (‾*x* ± *s*) was used for measurement data; *P* < 0.05 indicated that the difference was statistically significant.

## 3. Experimental Results and Observations

In this section, a detailed description of various experimental results and observations is provided with sufficient detail which enables every reader to fully understand the operational methodology of the proposed approach. For this purpose, a retrospective study or experiment was conducted on 150 patients with hypertensive intracerebral hemorrhage in the hospital specifically from January 2019 to January 2020. According to the nursing strategy, patients were divided into experimental (*n* = 75) and control groups (*n* = 75), respectively. The control group adopted routine nursing mode, whereas the experimental group adopted cluster nursing mode. The treatment compliance of patients in the experimental group was 86.67%, while that in the control group was 73.33% (*P* < 0.05). The total incidence of postoperative complications in the experimental group was 3.2%, which was lower than 25% in the control group (*P* < 0.05). The motor function score of the experimental group was better than that of the control group (*P* < 0.05). The application of cluster nursing in postoperative patients with hypertensive intracerebral hemorrhage is feasible, and its nursing effect is significant, which can not only reduce the incidence of postoperative complications but also improve patients' compliance and quality of life. It has good application value.

### 3.1. Patients' Compliance with Treatment

The treatment compliance rate of patients in the experimental group was significantly better than that in the control group, and the compliance rates were 86.67% and 73.33%, respectively, and the difference between the two groups was statistically significant (*P* < 0.05, Table 1).

### 3.2. Incidence of Complications

The total incidence of postoperative complications in the experimental group was lower than that in the control group, which was 4% and 24%, respectively. To put it simply, there were 4 cases of pulmonary infection, 6 cases of intestinal dysfunction, 5 cases of bedsore, 3 cases of DVT in the control group, 2 cases of intestinal dysfunction, and 1 case of bedsore in the experimental group. There was a significant difference in the incidence of complications between the two groups (*P* < 0.05, Table 2).

### 3.3. Motor Function Score

Before nursing, there was no significant difference in Fugl-Meyer score between the two groups, but after nursing, the Fugl-Meyer score of the two groups was higher than that before nursing, and the Fugl-Meyer score of the experimental group was higher than that of the control group.

After nursing, the Fugl-Meyer score of the two groups was higher than that before nursing, and the Fugl-Meyer score of the experimental group was higher than that of the control group, and the difference was statistically significant (*P* < 0.05, Table 3).

## 4. Discussion

Hypertensive intracerebral hemorrhage is a common neurological condition caused by arterial rupture and hemorrhage in the brain parenchyma of patients with hypertension or cerebral atherosclerosis. It is more common in men over 50 years old and has the characteristics of acute and serious illness, and the fatality rate is very high [9]. Postoperative hypertensive intracerebral hemorrhage may lead to complications such as pulmonary infection and deep venous thrombosis, with a high disability rate, even if surgical treatment can inhibit the development of cerebral hemorrhage; however, the occurrence of postoperative complications or the recurrence of cerebral hemorrhage will reduce patients' confidence in treatment, reduce patients' treatment compliance, and then lead to poor postoperative rehabilitation, poor improvement of motor function, and deterioration of patients' condition [10]. People pay more and more attention to hypertension as an important risk factor of cerebral hemorrhage in our country. The high fatality rate and disability rate have brought great challenges to the public health of our country; therefore, in order to reduce the mortality and disability rate caused by hypertensive intracerebral hemorrhage as much as possible, in addition to improving treatment techniques, high-quality nursing service is also very important. Effective nursing service can improve the self-confidence and enthusiasm of patients with hypertensive intracerebral hemorrhage and improve their treatment compliance, so as to improve the therapeutic effect and maximize the clinical symptoms, so as to improve the quality of life of patients with hypertensive intracerebral hemorrhage.

In order to ensure the treatment effect, the experimental group adopted the cluster nursing mode in this study. After the intervention, the treatment compliance of the patients was 86.67%, which was significantly higher than 73.33% of the control group. The incidence of postoperative complications in the experimental group was significantly lower than that in the control group, and the motor function score after the intervention was higher than that in the control group (*P* < 0.05). It shows that the nursing intervention under the guidance of the cluster nursing mode can reduce the pain of patients, build a more harmonious relationship between nurses and patients, and make the treatment compliance of patients higher. Compared with the traditional nursing mode, it can enhance the motor function of patients, promote the postoperative recovery of patients, and improve the quality of life of patients. We customized personalized treatment plans for patients from the aspects of respiratory intervention, posture intervention, nutritional intervention, psychological nursing, and quality control, so as to make patients feel professional nursing services, improve treatment compliance, better cooperate with nurses, and reduce the occurrence of postoperative bedsore, pulmonary infection, and deep venous thrombosis. The close relationship between mental disorders and chronic diseases has been widely accepted. Most patients with chronic diseases have psychological problems, which are not conducive to the recovery of the disease [11]. The cluster nursing mode attaches importance to psychological nursing, evaluates the psychological needs of patients, and then adopts targeted psychological nursing, communicates with patients more, understands the real thoughts of patients, establishes good feelings with patients, makes patients trust nursing staff, relieves patients' bad psychological emotions, and keeps them in a good psychological state.

However, this study excludes patients with serious diseases such as heart, lung, and kidney, history of cerebral infarction, and poor blood coagulation, so the sample size is small, and more samples will be included in the study. To sum up, cluster nursing can effectively improve the treatment compliance of postoperative patients with hypertensive intracerebral hemorrhage, improve patients' motor function, and reduce the incidence of postoperative complications, and it has been recognized by patients. It gives full play to the value of nursing service, provides a reference for nursing work, and can be popularized and applied in clinic.

## 5. Conclusion and Future Work

In this paper, cluster nursing was applied to the treatment of postoperative patients with hypertensive intracerebral hemorrhage. For this purpose, a retrospective study or experiment was conducted on 150 patients with hypertensive intracerebral hemorrhage in the hospital specifically from January 2019 to December 2020. According to the nursing strategy, patients were divided into experimental (*n* = 75) and control groups (*n* = 75), respectively. The control group adopted routine nursing mode, whereas the experimental group adopted cluster nursing mode. The treatment compliance of patients in the experimental group was 86.67%, while that in the control group was 73.33% (*P* < 0.05). The total incidence of postoperative complications in the experimental group was 3.2%, which was lower than 25% in the control group (*P* < 0.05). The motor function score of the experimental group was better than that of the control group (*P* < 0.05). The application of cluster nursing in postoperative patients with hypertensive intracerebral hemorrhage is feasible, and its nursing effect is significant, which can not only reduce the incidence of postoperative complications but also improve patients' compliance and quality of life. It has good application value.

In future, we are eager to investigate the effects of the proposed model on other well-known diseases in our country. Additionally, we will integrate the proposed model with other state-of-the-art models to develop a reliable and robust model for healthcare domain.

## Figures and Tables

**Table 1:** Changes of treatment compliance of patients in two groups after nursing intervention (*n* (%)).

Group	Number of cases	Good compliance	Moderate compliance	Poor compliance	Compliance rate (%)
Control group	75	35 (46.67)	20 (26.66)	20 (26.67)	73.33
Experimental group	75	50 (66.67)	15 (20)	10 (13.33)	86.67
*χ* ^2^	—	—	—	—	4.167
*P*	—	—	—	—	0.041

**Table 2:** Incidence of postoperative complications in two groups (*n* (%)).

Group	Number of cases	Pulmonary infection	Intestinal dysfunction	Bedsore	DVT	Incidence (%)
Control group	75	4 (5.33)	6 [8]	5 (6.67)	3 [4]	24
Experimental group	75	0	2 (2.67)	1 (1.33)	0	4
*χ* ^2^	—	—	—	—	—	17.564
*P*	—	—	—	—	—	<0.001

**Table 3:** Comparison of Fugl-Meyer scores between two groups before and after nursing (‾*x* ± *s*, points).

Group	Number of cases	Before nursing	After nursing	*t*	*P*
Control group	75	72.45 ± 6.25	82.36 ± 7.48	8.805	0.001
Experimental group	75	71.46 ± 6.43	91.56 ± 8.62	16.168	0.001
*t*	—	0.956	6.981	—	—
*P*	—	0.341	0.001	—	—

## Data Availability

The datasets used and analyzed during the current study are available from the corresponding author upon reasonable request.
